RETRACTED

# lncRNA-XLOC_012370 Promotes the Development of Pancreatic Cancer and Inactivates the NF-κB Pathway Through miR-140-5p

**DOI:** 10.3389/fonc.2020.620550

**Published:** 2021-02-23

**Authors:** Han-Xiao Nie, Ling Zhang, Tao He, Li Wang, Bai-Shun Wan, Xiao-Qian Wang, Feng Han

**Affiliations:** Department of Hepatopancreatobiliary Surgery, Henan Tumor Hospital Affiliated to Zhengzhou University, Zhengzhou, China

**Keywords:** pancreatic cancer, lncRNA-XLOC_012370, miR-140-5p, TLR4, NF-κB signal pathway

## Abstract

Pancreatic cancer is a high incidence, high degree of malignancy, and high mortality in the digestive system tumor. The incidence of pancreatic cancer in China has increased nearly six folds in the past 20 years, ranking fifth in the mortality rate of malignant tumors, so it is particularly important to actively explore clinical indicators with better diagnostic significance for pancreatic cancer. LncRNA performs an essential regulatory function in the occurrence, development, and metastasis of many kinds of tumors, playing both a carcinogenic role and a tumor suppressor gene. Here, we demonstrated the function and mechanism of LncRNA-XLOC_012370 in the development of pancreatic cancer. In our research, the abnormal upregulation of XLOC_012370 was observed in pancreatic cancer patients’ tumor tissues. XLOC_012370 was related to tumor stage, lymph node metastasis, and overall survival. Silencing of XLOC_012370 prevented the proliferation, migration, and invasion *via* the NF-κB signal pathway. Further, miR-140-5p was identified as the target and downstream of XLOC_012370 and involved in pancreatic cancer progression. *In vivo*, knockdown of XLOC_012370 inhibited tumor growth *via* the NF-κB signal pathway. In conclusion, lncRNA-XLOC_012370 is closely related to some malignant clinicopathological features and prognosis of pancreatic cancer. Thus the miR-140-5p/NF-κB signal pathway might represent a promising treatment strategy to combat pancreatic cancer.

## Introduction

The onset of pancreatic cancer is hidden, and its mortality ranks fourth among malignant tumors, and it is predicted that it will rise to second place by 2030 (1). Eighty five percent of the patients had local lymph node or distant organ metastasis at the time of diagnosis, which is the main reason for the poor clinical effect (2). Therefore, it is necessary to explore more pathogenesis of pancreatic cancer and explore new treatment methods.

LncRNA is a kind of endogenous RNA molecules whose length is larger than that of 200nt. Recent studies have shown that lncRNA may be involved in encoding short peptides (3). The synthesis of LncRNA is mainly formed by RNA polymerase II transcription, 5 ‘terminal addition, and 3’ polyadenylate cleavage. However, some lncRNAs are produced by RNA polymerase III and maintain the characteristics of non-polyadenosine acidification (4). LncRNA is located in the nucleus and cytoplasm, interacts with DNA, RNA, and proteins, and regulates gene expression before or after transcription. At present, people have realized that lncRNA is abnormally expressed in many diseases, including tumors (5). LncRNA MALAT1 is expressed in a variety of tissues and tumors, and it is also a lncRNA closely related to growth in pancreatic cancer (6, 7). Research showed that the high expression of MALAT1 in pancreatic ductal adenocarcinoma was related to poor prognosis. MALAT1 could bind to RNA binding protein HuR and down-regulate MALAT1, which promoted the post-transcriptional regulation of TIA-1 and inhibits autophagy (7). In addition, MALAT1 can competitively combine with miR-217 to regulate Kras level and induce the proliferation of pancreatic cancer cells (8). Gas5 is a lncRNA closely related to cell cycle and cell proliferation. Lu et al. found that Gas5 was significantly decreased in pancreatic tumor tissues, while the expression of Gas5 in pancreatic cancer cell lines was also considerably downregulation, suggesting that Gas5 is closely related to the occurrence of pancreatic cancer. Force expression of Gas5 significantly blocked PANC-1 cells development; after inhibiting the expression of Gas5 by RNA interference, the number of cells of G0/G1 phase decreased, and more cells enter in S phase, suggesting that Gas5 can regulate the cell cycle of pancreatic cancer cells and inhibit the invasion of cancer cells (9).

RETRACTED

Since the discovery of the NF-κB transcription factor in 1986, after long-term research, researchers have had a relatively complete understanding of its composition and regulation (10). The process of the NF-κB signal pathway eventually leads to the expression of different genes regulated by it, which plays different functions of inflammation and immunity, but the signal intensity of NF-κB needs to be maintained in a reasonable range. Otherwise, it will lead to abnormal gene expression and eventually lead to the occurrence of various diseases (11). The feedback regulation of IkB molecules to the NF-κB signal pathway is a widely recognized regulation mode. The word feedback regulation is used because the expression of IkBx and IkB ϵ molecules is regulated by the NF-κB signal pathway. That is, activated NF-κB signal can increase the expression of IkB molecules, while the expression of the latter is negatively fed back to the NF-κB signal pathway to reduce its expression (12). The existing experimental data have fully shown that inhibition of the NF-κB signal pathway can inhibit tumor proliferation and promote tumor cell apoptosis, so it is a hot spot in tumor medicine to develop inhibitors for tumor therapy. So far, more than 700 kinds of NF-κB inhibitors have been found. Bortezomib is a 26S proteasome inhibitor, and there is also evidence that it can inhibit the degradation of IkB molecules and further inhibit the expression of NF-κB signal in cells, while Wissniowski et al. suggested that pancreatic tumor cells with high secretion are more sensitive to Bortezomib (13). Curcumin was another drug that has been reported to inhibit the activity of the NF-κB signaling pathway. Cell experiments have given evidence of its inhibition of pancreatic tumor cells (14).

RETRACTED

Here, we detected the level of XLOC_012370 in pancreatic cancer patients’ tissues and clinical significance. Then we explored the function of XLOC_012370 in pancreatic cancer cell development. Meanwhile, we identified the paired miRNA and confirmed the relationship between XLOC_012370 and miRNA.

## Method and Materials

### Clinical Samples

The tumor samples were collected from 30 pancreatic cancer patients at Henan Tumor Hospital Affiliated to Zhengzhou University. After the collection, the tissues were immediately stored in liquid nitrogen and then kept at −80°C for further use. Experimental procedures were accomplished in accordance with the guidelines released by the Ethics Committee of Henan Tumor Hospital Affiliated to Zhengzhou University. Signed written informed consent was obtained from each patient.

The animal study was reviewed and approved by Henan Tumor Hospital Affiliated to Zhengzhou University.

### Cell Culture and Treatment

Human pancreatic cancer cell lines (PACN-1 and BxPC-3) were purchased from the Science Cell Laboratory. Cells were cultured in PRIM 1640 (Thermo-Life, United States) with 10% FBS (Thermo Fisher, USA) and 100 μl/ml penicillin and streptomycin (Beyotime, China) and placed at 37°C with 5% CO_2_.

Prior to transfection, the cells covered approximately 60% of the plates, with the culture medium in each well replaced with PRIM 1640 without serum, penicillin, or streptomycin for 2-h culture. Next, 1.5 ml Opti-MEM was added to the cells and pre-heated in an incubator. The plasmids, including si-miR-140-5p, miR-140-5p mimic, and negative control (NC), purchased from Shanghai Novo Biotechnology Co., Ltd. (Shanghai, China), and sh-XLOC_012370, sh-NC were purchased from Shanghai Genechem Co., Ltd. (Shanghai, China), Opti-MEM, and Lipofectamine^®^ 2000 transfection reagent (Invitrogen Inc., Carlsbad, CA, USA) were mixed in an even manner and permitted to stand for 5 min. The mixture was then added to the cells culture medium and mixed evenly. After incubation for 24 h, a fresh culture medium was added to the cells. After transfection for 48 h, the cells were detached with trypsin and collected for later experiments.

RETRACTED

### Western Blot

After RIPA cleavage, we extracted total protein and measured with the BCA method. After quantitative denaturation, protein electrophoresis membrane transfer and blocked. The first incubation and second incubation were carried out according to the operation steps. The expression of the protein was expressed by the gray value.

### Real Time-PCR

Total RNA was isolated from cells according to a standard protocol. And then, the purity and concentration of RNA were detected, and all the samples were converted into cDNA using a reverse transcription kit. We used SYBR Green (Thermo Fisher Scientific) system to perform the qRT-PCR. Data were analyzed by GraphPad 7.

### CCK8 Assay

The cells in the logarithmic growth phase were collected by centrifugation after trypsin digestion and resuscitated, and the cell count has adjusted to 2 × 10^4^/ml. The prepared cell suspension was gently mixed while adding a 96-well plate with 100 μl per well, and the inoculated cell culture plate was put into the incubator overnight, while the blank control group only added medium without cells, and 6 multiple holes were set up in each group to take the average value. The cell viability was measured by the CCK8 method after 24, 48, and 72 h, and 10 μl CCK8 solution was added to each well in different time groups and control groups, and the incubator was incubated for about 2 h. The absorbance (A) value of wells was detected at 450 nm of the enzyme labeling instrument.

### Matrigel Invasion Assay

In this experiment, a transwell chamber with a diameter of 6.5 mm and a pore size of 8 μm was selected; 0.25% trypsin was used to digest the cells in the logarithmic phase, resuscitated with 1640 basic medium and adjusted the cell density to 5 × 10^5^ ml; 100 μl cell suspension was added to the upper Transwell chamber, 500 μl 1640 medium (5% FBS) was added to the lower transwell chamber, and cultured for 24 h in the CO2 incubator; the transwell chamber was removed, the culture medium was absorbed, and the PBS was washed for three times. Twenty minutes; the discarded fixing solution was fixed in 4% paraformaldehyde solution, PBS shaker was washed for 10 min, crystal violet was dyed at room temperature for 10 min; PBS and washed twice, 5 min; each time, the cells on the upper surface of the chamber were wiped off with skimmed cotton, and five visual fields were photographed and counted under the microscope for follow-up statistics and analysis.

RETRACTED

### Statistical Analysis

All values are expressed as the mean ± SEM. Statistical significances were measured by Student’s t-test and ANOVA. A two-tailed value of P < 0.05 was indicated as a statistically significant difference. Data statistics were used the Prism 7.0.

## Results

### XLOC_012370 Was Up-Regulated in Pancreatic Cancer

Firstly, we used bioinformatics to analyze the differentially expressed lncRNA genes in tumor tissues and adjacent tissues from pancreatic cancer patients (**Figure 1A**). According to microarray data, serious of significantly up-regulated lncRNAs were found in tumor tissues and corresponding adjacent normal tissues. Among these up-regulated lncRNAs, XLOC_012370 was considerably higher than other lncRNAs. To explore the function of XLOC_012370 in pancreatic cancer, we collected 30 pancreatic patients’ tumor tissues and adjacent normal tissues. We observed that XLOC_012370 was significantly increased in tumor tissues (**Figure 1B**). Meanwhile, the expression of XLOC_012370 in the plasma from pancreatic patients and healthy volunteers were detected. We also observed the increased level in pancreatic patients (**Figure 1C**).

**Figure 1:** LncRNA XLOC_012370 was upregulation in pancreatic cancer tissues. **(A)** ChIP analysis of tumor samples. Tumor tissues and adjacent normal tissues were collected from pancreatic cancer patients. **(B)** The expression of lncRNA XLOC_012370 in tumor tissues and adjacent normal tissues were detected by RT-PCR. n=30, *P < 0.05. **(C)** The expression of lncRNA XLOC_012370 in plasma from pancreatic cancer patients and healthy volunteers were detected by RT-PCR. n=30, *P < 0.05.

### XLOC_012370 Is Associated with Clinicopathologic Characteristics and Prognosis of Pancreatic Cancer Patients

We found that the expression of XLOC_012370 was higher in stage II and stage III pancreatic cancer patients (**Figure 2A**). Meanwhile, we observed that the expression of XLOC_012370 was associated with lymph node metastasis. With the increase of the degree and extent of lymph node involvement, the expression of XLOC_012370 was also increased (**Figure 2B**). Further, we found that the overall survival of pancreatic patients with low expression of XLOC_012370 was significantly higher than pancreatic patients with high expression of XLOC_012370 (**Figure 2C**). In summary, XLOC_012370 was associated with clinical features of pancreatic cancer

**Figure 2:** Associations between XLOC_012370, clinicopathologic characteristics, and prognosis after surgery. **(A)** XLOC_012370 expression in different TNM stages of pancreatic cancer, stages I, II, and III (n = 13, n = 9, and n = 8, respectively). *P < 0.05. **(B)** XLOC_012370 expression in the lymph node metastasis-N0 group (N0, n = 7), -N1 group (N1, n = 9), and -N2 group (N2, n = 6). *P < 0.05. **(C)** Overall survival curve of the high-level and low-level group divided by XLOC_012370 expression. *P < 0.05.

RETRACTED

### Silencing of XLOC_012370 Prevents Development in Pancreatic Cancer Cells

Then we constructed shRNA for silencing XLOC_012370 gene expression. The transfection efficiency of shRNA was identified by RT-PCR (**Figure 3A**). Then we performed a CCK8 assay for cellular viability. As **Figure 3B** shown, sh-XLOC_012370 significantly inhibited the cellular viability in BXPC3 and PANC-1 cells. The clone formation capacity of BXPC3 and PANC-1 cells was assessed by the clone formation assay, which performed inhibition function by sh-XLOC_012370 (**Figure 3C**). EdU incorporation of cancer pancreatic cancer cells was conducted to explore cell proliferation rates. The proliferation potential of the BXPC3 and PANC-1 cells was significantly reduced after sh-XLOC_012370 transfection (**Figure 3D**). Wound healing and transwell migration assay results revealed that sh-XLOC_012370 inhibited the migration ability of pancreatic cancer cell lines (**Figures 3E, F**). XLOC_012370 knockdown inhibited tumor cell invasion, as demonstrated by a transwell invasion assay (**Figure 3F**). Further, the protein expression of the NF-κB signaling pathway was analyzed by immunoblot assay. As we observed, XLOC_012370 knockdown prevented phosphorylation of P65 and up-regulated IκBα (**Figure 3G**). Taken together, knockdown of XLOC_012370 would prevent the development of pancreatic cancer cells *via* inactivating the NF-κB signaling pathway.

**Figure 3:** Silencing of XLOC_012370 promotes proliferation, migration, and invasion in PANC-1 and BxPC-3 cells. **(A)** Efficiencies of XLOC_012370 knockdown in PANC-1 and BxPC-3 cells were detected by qRT-PCR assays. n=5, *P < 0.05. **(B)** The cell viability of sh- XLOC_012370-transfected PANC-1 and BxPC-3 cells were detected by CCK-8 assays. n=6, *P<0.05. **(C)** Effect of XLOC_012370 knockdown on colony formation was counted in PANC-1 and BxPC-3 cells. n=4, *P < 0.05. **(D)** Representative images and histogram analysis of EdU assays after XLOC_012370 knockdown in PANC-1 and BxPC-3 cells. n=3, *P <0.05. **(E)** Wound healing assays after XLOC_012370 knockdown in PANC-1 and BxPC-3 cells. n=3, *P < 0.05. **(F)** Representative images and histogram analysis of transwell assays after XLOC_012370 knockdown in PANC-1 and BxPC-3 cells. n=4, *P < 0.05. **(G)** The protein level of IκBα, P65, and p-P65 were detected in PANC-1 cells.

### MiR-140-5p Is Downstream of XLOC_012370 in Pancreatic Cancer

First, multiple bioinformatics prediction websites analysis miR-140-5p was a potential target of XLOC_012370 (**Figure 4A**). Endogenous XLOC_012370 pull-down by AGO2 was enriched in cells transfected with miR-140-5p, revealing the direct binding of XLOC_012370 with miR-140-5p (**Figure 4B**). Further, luciferase assay performed that miR-140-5p could interact with XLOC_012370 and miR-140-5p (**Figure 4C**). We also found that XLOC_012370 and miR-140-5p have a negative correlation (**Figure 4D**). Colocalization analysis of miR-140-5p and XLOC_012370 in PANC-1 cells was confirmed by FISH staining (**Figure 4E**).

RETRACTED

**Figure 4:** LncRNA XLOC_012370 interacts with miR-140-5p. **(A)** Bioinformatic target prediction was performed with three online tools. **(B)** Binding situation between XLOC_012370 and miR-140-5p verified using RNA pull-down. n=3, *P < 0.05, **P < 0.01. **(C)** Luciferase assay was performed in the relationship between XLOC_012370 and miR-140-5p. n=3, *P < 0.05. **(D)** Pearson analysis of the correlation of miR‐140‐5p with XLOC_012370 expression in tumor tissues. n=30. **(E)** Co-localization between XLOC_012370 and miR-140-5p was revealed by fluorescence *in situ* hybridization. n.s. means not significant.

### Silencing of XLOC_012370 Prevents Tumor Progression by Regulating miR-140-5p In Vitro

After sh-XLOC_012370 vector and si-miR-140-5p transfection, the cells were performed with CCK8 assay. The results showed that the decreased cell viability induced by sh-XLOC_012370 was inhibited by si-miR-140-5p treatment (**Figure 5A**). Clone formation assay performed that si-miR-140-5p blocked the function of sh-XLOC_012370 in BXPC3 and PANC-1 cells (**Figure 5B**). The proliferation potential of the pancreatic cancer cells was significantly prevented by sh-XLOC_012370, which was reversed by si-miR-140-5p (**Figure 5C**). Wound healing and transwell assay results revealed that si-miR-140-5p inhibition remitted the migration and invasion function of sh-XLOC_012370 in pancreatic cancer cell lines (**Figures 5D, E**). Further, it forced the decreased expression of the XLOC_012370 inactivated NF-κB signal pathway, which was inhibited by si-miR-140-5p (**Figure 5F**). In short, XLOC_012370 was involved in regulating the development of pancreatic cancer *via* regulating miR-140-5p.

**Figure 5:** XLOC_012370 regulates tumor progression *via* targeting miR-140-5p. **(A)** The cell viability of PANC-1 and BxPC-3 cells were detected by CCK-8 assays. n=5, *P < 0.05, ^#^ *P* < 0.05. **(B)** Colony formation was counted in PANC-1 and BxPC-3 cells. n=3, *P < 0.05, ^#^ *P* < 0.05. **(C)** Representative images and histogram analysis of EdU assays in PANC-1 and BxPC-3 cells. n=3, *P < 0.05, ^#^ *P* < 0.05. **(D)** Wound healing assays in PANC-1 and BxPC-3 cells. n=3, *P < 0.05, ^#^ *P* < 0.05. **(E)** Representative images and histogram analysis of transwell assays in PANC-1 and BxPC-3 cells. n=3, *P < 0.05, ^#^ *P* < 0.05. **(F)** The protein level of IκBα, P65, and p-P65 was detected in PANC-1 cells. n=4, *P < 0.05, ^#^ *P* < 0.05, **P < 0.01.

RETRACTED

### Forced Down-Regulation of XLOC_012370 Promotes Tumorigenicity In Vivo

To further explore the function of XLOC_012370 in pancreatic cancer, we set up a xenograft nude mice model. sh-XLOC_012370/sh-NC-PANC-1 cells were subcutaneously injected into nude mice, and we measured tumor volume. Kaplan–Meier survival curve of mice, monitored for 30 days (**Figure 6A**). sh-XLOC_012370 significantly reduced tumor volume and weight (**Figures 6B, D**). The tumor tissue was sectioned for immunohistochemical staining. As **Figure 6E** shown, the Ki-67 staining performed that sh-XLOC_012370 significantly inhibited the proliferation of tumors, which was consistent with the results *in vitro*. Then the collected tumor tissues for P65 and IκBα detection. Similar to the results *in vitro*, we found the induced IκBα expression and decreased p-P65 (**Figure 6F**). The above results show that the XLOC_012370 knockdown would prevent tumor development and metastasis *in vivo* and *vitro.*

**Figure 6:** Sh-XLOC_012370 prevents tumor growth *in vivo*. **(A)** Kaplan–Meimer survival curve of tumor-bearing nude mice. *P < 0.05. **(B, C)** Tumor volume and tumor weight were analyzed. n=7, *P < 0.05. **(D)** Tumors removed from the mice 30 days, respectively n=7. **(E)** Representative image of ki-67 staining. **(F)** The protein level of IκBα, P65, and p-P65 were detected in the tumor. n=6, *P < 0.05.

## Discussion

Many research has shown that non-coding RNA plays an essential role in the occurrence and development of pancreatic cancer. The biological functions of lncRNAs include epigenetic regulation, transcriptional regulation, post-transcriptional regulation, miRNA regulation, cell differentiation, and development (3). One of its essential mechanisms is to regulate the selective expression of related coding genes around it. Urothelial carcinoma-associated 1 (UCA1) was first found in transitional cell carcinoma of the bladder, which plays an essential role in tumorigenesis, development, and drug resistance (15, 16). Chen et al. showed that the expression level of UCA1 in pancreatic cancer tissues was significantly increased, and its expression level was positively correlated with tumor size, clinical stage, CA19-9 level, and total survival time. Further inhibition of UCA1 expression in BXPC3 cells by RNA interference can effectively inhibit tumor cell proliferation and induce tumor cell apoptosis (17). The expression of UCA1 is negatively correlated with the tumor suppressor gene p27. UCA1 can promote the proliferation of tumor cells by inhibiting the expression of p27 and its downstream genes. UCA1 can also promote the migration and invasion of pancreatic cancer by regulating matrix metalloproteinases. Zhang et al. also proved that the expression of UCA1 is up-regulated in human pancreatic cancer and confirmed for the first time that UCA1 might promote the progression of pancreatic cancer through the Hippo signal transduction pathway (16). Overexpression of UCA1 inhibits YAP phosphorylation and increases YAP expression. UCA1 interacts with MOB1, Lats1, and YAP to form protective complexes, inhibit their phosphorylation, and promote the transfer of YAP to the nucleus, thus enabling the malignant phenotype and carcinogenic function of pancreatic cancer cells (18). In the study of the carcinogenic mechanism of PVT1, it was found that PVT1 and myc genes were close to and co-amplified. In Burkett’s lymphoma, breast cancer, and lung cancer, and other solid tumors, it has been confirmed that the increased expression of PVT1 can increase the expression of carcinogen myc. There was also a significant difference in the level of PVT1 in saliva between patients with pancreatic cancer and normal controls (19). Here, we found the increased expression of XLOC_012370 in pancreatic cancer tumor tissues. The silencing of XLOC_012370 could inhibit the progression of pancreatic cancer.

RETRACTED

Recently, studies have found that there are many abnormal expressions of miRNAs in pancreatic cancer, some of which are found in precancerous pancreatic lesions (20). Some are found in pancreatic cancer tissue specimens, and some are found in the serum of pancreatic cancer patients (21, 22). Szafranska et al. found that 94 miRNAs were abnormally expressed in human normal pancreatic tissue, pancreatic cancer cell line, chronic pancreatitis tissue, and pancreatic cancer tissue (23, 24). Therefore, the researchers believe that these differentially expressed miRNAs may provide new clues for the study of pancreatic cancer, and some studies have shown that miRNAs are related to apoptosis, invasion, and metastasis of cancer. For example, overexpression of miR-10a can inhibit HOXA1 and cause local invasion of pancreatic cancer (25). Reducing the expression of miR-125a-5p will inhibit the proliferation and cell cycle of pancreatic tumors and promote the apoptosis of early cancer cells (26). Here, we found that miR-140-5p could interact with XLOC_012370 and involve in XLOC_012370, regulating the progression of pancreatic cancer.

RETRACTED

In recent years, lncRNA, which was once regarded as transcriptional “noise,” has gradually become a research hotspot. However, at present, most of the studies on lncRNA are at the primary level, such as discovering new lncRNA and exploring its abnormal expression in tumors, and its specific mechanism in tumors still needs to be further discussed (27). In addition, due to the hidden incidence of pancreatic cancer, there are no apparent symptoms in the early stage. With the progress of detection methods, lncRNA can be obtained from both body fluid and tissue samples of pancreatic cancer, which provides us with good technical conditions for the study of pancreatic cancer. Many lncRNA has been preliminarily confirmed in pancreatic cancer, but lncRNA also has some problems such as poor specificity and unclear mechanism of action, which is still a long way from clinical application. In the future, the related research on lncRNA in pancreatic cancer should also focus on the process of pancreatic cancer proliferation, metastasis, drug resistance, early diagnosis, prognosis and curative effect prediction, biomarker screening, and so on. However, it is undeniable that lncRNA has great potential in the occurrence and development, early diagnosis, prognosis, and prognosis of pancreatic cancer. Understanding its mechanism will help to provide a new direction for finding new targets for the treatment of pancreatic cancer.

## Conclusion

Here, we identified that XLOC_012370 was increased in pancreatic cancer tumor tissues. The level of XLOC_012370 was related to the clinicopathologic characteristics of pancreatic cancer patients. The silencing of XLOC_012370 significantly suppressed pancreatic cancer cell progression. Further, we revealed that XLOC_012370 promoted tumor progression *via* the NF-κB signal pathway by regulating miR-140-5p.

## Data Availability Statement

The original contributions presented in the study are included in the article/supplementary material. Further inquiries can be directed to the corresponding author.

## Ethics Statement

The studies involving human participants were reviewed and approved by Henan Tumor Hospital Affiliated to Zhengzhou University. The patients/participants provided their written informed consent to participate in this study. The animal study was reviewed and approved by Henan Tumor Hospital Affiliated to Zhengzhou University.

## Author Contributions

HXN and LZ performed the majority of experiments and analyzed the data. LW and BSW performed the molecular investigations. TH designed and coordinated the research. XQW and FH wrote the paper. All authors contributed to the article and approved the submitted version.

RETRACTED

## Conflict of Interest

The authors declare that the research was conducted in the absence of any commercial or financial relationships that could be construed as a potential conflict of interest.
